# Transient activation of the PI3K/Akt pathway promotes Newcastle disease virus replication and enhances anti-apoptotic signaling responses

**DOI:** 10.18632/oncotarget.15796

**Published:** 2017-03-01

**Authors:** Yinfeng Kang, Runyu Yuan, Xiaqiong Zhao, Bin Xiang, Shimin Gao, Pei Gao, Xu Dai, Minsha Feng, Yanling Li, Peng Xie, Yulian Li, Xiaoyi Gao, Tao Ren

**Affiliations:** ^1^ Key Laboratory of Zoonosis Prevention and Control of Guangdong Province, College of Veterinary Medicine, South China Agricultural University, Guangzhou, 510642, China; ^2^ State Key Laboratory of Oncology in South China, Collaborative Innovation Center for Cancer Medicine, Department of Experimental Research, Sun Yat-sen University Cancer Center, Guangzhou, 510060, China; ^3^ Key Laboratory of Animal Vaccine Development, Ministry of Agriculture, Guangzhou, 510642, China; ^4^ Key Laboratory for Repository and Application of Pathogenic Microbiology, Research Center for Pathogens Detection Technology of Emerging Infectious Diseases, Guangdong Provincial Center for Disease Control and Prevention, Guangzhou, 510300, China; ^5^ College of Animal Science and Technology, Shanxi Agricultural University, Jinzhong, 030800, China

**Keywords:** Newcastle disease virus, PI3K/Akt, replication, apoptosis, cell survival

## Abstract

Viral infection activates a host's cellular phosphatidylinositol 3-kinase (PI3K)/Akt signaling pathway, which is involved in cell differentiation, growth, survival, and apoptosis. To elucidate molecular mechanisms in the pathogenesis of Newcastle disease virus (NDV), we demonstrated that NDV transiently activates the PI3K/Akt pathway in chicken cells at an early phase of infection. Its activation was observed as early as 15 min post-infection and gradually weakened after 24 h. Incubating cells with a PI3K inhibitor, LY294002 or wortmannin, prior to NDV infection decreased NDV progeny yields and suppressed Akt phosphorylation at early times post-infection. Akt activation is triggered by NDV-GM or NDV-F48E9 and is abolished by methyl β-cyclodextrin and chlorpromazine. Treatment following NDV-La Sota infection had no obvious effect. However, inhibiting PI3K activation promoted apoptotic responses during an early stage of NDV infection. The pan caspase inhibitor ZVAD-FMK mitigated the reduction in Akt phosphorylation by inhibiting PI3K activation, which indicates the signaling pathway promotes cell survival and, in turn, facilitates viral replication. By suppressing premature apoptosis upon NDV infection, the PI3K/Akt pathway enhances the anti-apoptotic response.

## INTRODUCTION

Newcastle disease virus (NDV) is a negative-sense, single-stranded, RNA virus of the *Paramyxoviridae* family with a promising oncolytic agent against tumor cells in Phase I clinical studies [1, 2]. The NDV genome encodes at least six structural proteins: the nucleocapsid protein (NP), matrix protein (M), phosphoprotein (P), fusion protein (F), hemagglutinin–neuraminidase protein (HN), and large polymerase protein (L) [3]. The *P* gene additionally encodes the three proteins P, V, and W by way of RNA editing [4]. Earlier research has shown that the V and W proteins promote NDV replication and pathogenicity [5]. NDV binds to the sialic acid of cell surface receptors via the HN protein and, by analogy, to other paramyxoviruses’ pH-independent mechanisms mediating the membrane by F protein's direct integration into host cells [6]. NDV enters a host's infected cells via the pH-dependent mechanisms of receptor-mediated endocytosis, in which the virus envelope fuses with the cellular membrane, as also occurs with viruses in Togaviridae, Rhabdoviridae, Orthomyxoviridae, Flavivirus, and with false virus [7, 8].

The phosphatidylinositol 3-kinase (PI3K)/Akt signaling pathway stimulates a variety of cells’ activities, including growth, proliferation, survival, migration, metabolism, and apoptosis [9]. When PI3K is activated by G protein-coupled receptors and tyrosine kinase receptors, phosphatidylinositol 3,4-bisphosphate phosphorylates 3,4,5-tris phosphatidylinositol phosphate, which binds and recruits Akt to the cellular membrane. Thr308 and Ser473 are phosphorylated by PDK1 and mTORC2, respectively, and this in turn activates the Akt and downstream signaling pathways [10, 11]. Various viruses, including the hepatitis C virus, vaccinia virus, avian leukemia virus, human cytomegalovirus, coxsackie B3 virus, and Sendai virus activate the PI3K/Akt signaling pathway by attaching to the host cell membrane surface. This activates virus internalization and endosomal sorting processes that facilitate viral replication [12]. Following the invasion of host cells, influenza virus A (H5N1) activates PI3K/Akt via NS1 protein, which promotes viral replication and inhibits apoptosis [13]. In the early stages of infection, the respiratory syncytial virus activates the PI3K/Akt pathway, Mdm-2 upregulation, and P53 degradation, thereby promoting cell survival [14]. Though PI3K/Akt promotes most viral replication, cell survival, and proliferation, it suppresses the replication of the hepatitis B virus [15]. No studies have reported whether NDV activates the PI3K/Akt signaling pathway.

In NDV-infected cells or animals, especially in the early stages of infection, NDV can trigger apoptosis, thereby inhibiting proliferation. Specifically, the activation of caspase 3, caspase 8, and caspase 9 can induce apoptosis and increase the activity of members of the Bcl-2 family, including Bcl-2, Bcl-xL, Bax, and Bad [12]. Although many viruses activate the PI3K/Akt signaling pathway to promote cell survival and inhibit apoptosis, the relationship of the pathway and NDV remains unexplored. To better understand the mechanism of molecule pathogenesis in NDV infection, we used the CEF and DF-1 cell models to investigate the interaction among NDV, the PI3K/Akt signaling pathway, and apoptosis.

## RESULTS

### Transient activation of Akt by NDV

To determine whether NDV could affect the PI3K/Akt pathway, we infected CEF and DF-1 cells with NDV strains GM, La Sota, or F48E9 at an MOI of 1, and analyzed Akt at different time points for 48 h after infection. NDV did not affect the overall protein level of Akt in infected cells, but it induced the phosphorylation of Akt at serine 473 between 2 and 24 h postinfection (hpi). By 24 hpi, the induction of Akt phosphorylation had declined and gradually become visible again (Figure 1A). This suppression of Akt phosphorylation by NDV was even more pronounced at 48 hpi. Since the induction of Akt phosphorylation became visible at 2 hpi in infected cells, we investigated the induction of Akt phosphorylation at earlier time points in response to NDV infection. Akt phosphorylation at serine 473 became detectable as early as 15 min postinfection (mpi) (Figure 1B).

**Figure 1:** Transient activation of Akt by NDV (**A**) CEF cells were infected with NDV-GM, NDV-La Sota, or NDV-F48E9 at an MOI of 1 for 0, 2, 4, 6, 9, 12, 24, 36, and 48 h. Cells were analyzed for Akt phosphorylation at serine 473 (pAkt 473), and overall Akt by western blot. (**B**) Cells were infected with NDV-GM, NDV-La Sota, or NDV-F48E9 at an MOI of 1, and cell lysates were harvested at 15 min intervals until 2 hpi. Akt phosphorylation at serine 473 (pAkt 473) was analyzed by western blot.

To verify whether the phosphorylation of Akt in CEF and DF-1 cells was PI3K dependent or independent following infection with NDV, the specific PI3K inhibitors LY294002 (10 and 20 μM) and wortmannin (0.2 and 1 μM) were incubated for 1 h prior to infection with NDV. Cells were harvested and lysed at 1 hpi, and then subjected to immunoblot analysis in order to detect Akt phosphorylation. NDV infection increased the induction of Akt phosphorylation, though the LY294002 or wortmannin pretreatment inhibited NDV from inducing Akt phosphorylation, yet without altering Akt's overall protein level in infected cells (Figure 2). Such results demonstrated that NDV's induction of Akt's phosphorylation is involved in the PI3K-dependent molecular mechanism.

**Figure 2:** Inhibition of NDV-induced Akt phosphorylation following treatment with the PI3K inhibitor LY294002 (LY) (**A**) or wortmannin (wort) (**B**). CEF cells were preincubated with LY294002 (10 and 20 μM) or wort (0.2 μM and 1 μM) for 1 h, and subsequently infected with NDV-GM (a), NDV-La Sota (b), or NDV-F48E9 (c) at an MOI of 1. After 1 h, cell lysates were harvested for pAkt (Ser 473) and total Akt detection was analyzed by western blot.

### Early endocytotic events of NDV infection involved in activating the PI3K/Akt pathway

NDV can enter infected cells via either receptor-mediated endocytosis or the activation of the fusion protein, provided that the interaction of viral glycoproteins with the receptor is in the early stages of the NDV life cycle [6, 7]. To determine whether these entry mechanisms are involved in inducing Akt phosphorylation by NDV infection, we analyzed the effect of two inhibitors of clathrin- or caveolae-dependent endocytosis. Chlorpromazine is a cationic amphiphilic compound that at once prevents the recycling of clathrin and blocks clathrin-dependent endocytosis [16]. The sterol-binding drug MβCD that sequesters cholesterol also depletes cholesterol in the plasma membrane [17]. We investigated the effects of both chlorpromazine and MβCD on the activation of Akt phosphorylation induced by NDV infection. Pretreating cells with various concentrations of chlorpromazine decreased Akt phosphorylation induced by GM and F48E9 infection, but had no effect on Akt phosphorylation expression induced by the La Sota strain (Figure 3). Furthermore, preincubating cells with various concentrations of MβCD diminished the induction of Akt phosphorylation induced by GM and F48E9 infection, but not induced by the La Sota strain. Those results suggest that Akt activation induced by NDV infection via clathrin- and caveolae-mediated endocytosis is dependent on a very early event during NDV entry.

**Figure 3:** Early events of endocytosis on NDV infection involved in PI3K/Akt pathway activation CEF cells were preincubated with chlorpromazine (5–50 μM) (**A**) or methyl β-cyclodextrin (1–10 mM) (**B**) for 1 h and subsequently infected with NDV-GM (a), NDV-La Sota (b), or NDV-F48E9 (c) at an MOI of 1. After 1 h, cell lysates were harvested for pAkt (Ser 473), and total Akt detection was analyzed by western blot.

Akt status triggered by NDV made Akt phosphorylation visible as early as 15 mpi, thereby indicating that the activation of PI3K/Akt signal transduction pathway is possibly involved in the interaction of NDV and its receptors at an early stage of viral infection. To validate that hypothesis, we infected CEF cells with UV light-irradiated NDV and harvested cell lysates at 1, 2, and 12 hpi for immunoblot analysis with the anti-phospho-Akt antibodies. UV light irradiation did not affect the interaction of NDV and its receptors, but it inhibited viral genomic RNA replication and damaged the NDV life cycle soon after NDV entry. P protein with UV light-irradiated NDV was reduced compared to cells infected by only NDV at 1, 2, and 12 hpi (Figure 4). However, the UV treatment of CEF cells did not decrease Akt phosphorylation or its overall protein level at serine 473 at those time points. This suggests that an initial event during NDV entry triggered the activation of Akt, and the activation of Akt phosphorylation was not required for virus replication.

**Figure 4:** Effect of ultraviolet (UV) irradiation on Akt activation by NDV NDV-GM with and without UV irradiation for 30 min were used to infect CEF cells, which were harvested and lysed at 0, 1, 2, and 12 hpi to detect pAkt (Ser 473) and NDV phosphoprotein (P).

### Inhibition of the PI3K/Akt pathway reduces viral replication

To evaluate whether activated Akt triggered by NDV was critical for virus replication, we detected and quantified the virus titers with or without incubation in the specific PI3K inhibitor LY294002 (20 μM) via plaque assay. CEF cells were pretreated with LY294002 for 1 h and infected with NDV-GM at an MOI of 1. Cell culture supernatants were harvested and quantified every 8 h for 64 hpi using plaque assay. To further investigate the role of Akt in NDV infection and rule out the possibility of reduced viral yields in infected cells due to the cytotoxic effect of the drugs, cell viability in the presence of either LY294002 or DMSO was first determined by MTT assay. Compared to the DMSO control treatment, LY294002 treatment had no apparent effect (0.2–4.9%) on cell viability at the time points indicated (Figure 5A). However, viral yields in the presence of specific PI3K inhibitor LY294002 was lower than non-LY294002-treated positive controls at 8 h to 64 h postinfection (Figure 5B). These results further indicate that the PI3K/Akt signaling pathway promotes NDV replication.

**Figure 5:** Inhibition of the PI3K/Akt signal transduction pathway decreases NDV titers (**A**) CEF cells were pretreated with DMSO or LY294002 (20 μM) for 1 h, and cell viability was measured and quantified by MTT cell proliferation assay at the time points indicated. (**B**) CEF cells were preincubated with LY294002 (20 μM) for 1 h, infected with NDV-GM at an MOI of 1, and cell culture media supernatant aliquots were harvested at 8-h intervals until 64 hpi. Virus titers in the cell supernatant were determined in CEFs via plaque assay. Data are representative of the results of three independent experiments; *p < 0.05, **p < 0.01 (*t* test).

### Suppression PI3K activity early in NDV life cycle inhibits viral progeny yields

To analyze at which time points PI3K activity occurred during the NDV life cycle, we preincubated CEF cells with either the specific PI3K inhibitor LY294002 (20 μM) or DMSO for 1 h at -60, -30, 0, 30, 60, 120, and 240 mpi, respectively. At 24 hpi, the supernatants were harvested and quantified by standard plaque assay in order to calculate viral progeny yields. Compared to the DMSO control treatment, LY294002 inhibited viral progeny yields up to 60% at all timepoints except 240 mpi (Figure 6). Similarly, PI3K inhibitor wortmannin (1 μM) also suppressed virus replication at early time points of infection. These suggest that PI3K activity stimulates efficient replication of NDV early on in its life cycle.

**Figure 6:** Inhibition of the PI3K activity at the early, but not the later, phase of infection results in reduced titers of NDV progeny CEF cells were treated with LY294002 (20 μM) or DMSO starting at the indicated time points before and during infection with NDV-GM at an MOI of 1. At 24 hpi, virus titers were monitored by plaque assay. Data are representative of the results of three independent experiments, both performed in triplicate; ns: Not significant, *p < 0.05, **p < 0.01 (*t* test).

### Inhibition lysosomal acidification decreases Akt phosphorylation and NDV replication

To investigate whether inhibiting pattern recognition receptors such as Toll-like receptors (TLR) affects Akt phosphorylation and viral yields, we added the 4-aminoquinoline drug chloroquine (CQ) to infected cells. CQ can decrease lysosomal acidity, alter lysosomal permeability, inhibit TLR7 and TLR8 activity, and prevent the acidification of endosomes [18, 19]. CEF cells were pretreated for 1 h with increasing concentrations of lysosomal acidification inhibitor CQ (5, 10, 20, 50, and 100 μM). After NDV-GM infection at an MOI of 1, they were harvested for the detection of Akt phosphorylation by immunoblot analysis. Akt phosphorylation at serine 473, but not its overall protein level, gradually decreased with increasing concentrations of CQ (Figure 7A), which suggests that inhibiting lysosomal acidification in turn inhibits PI3K activity. Cells were also preincubated with various concentrations of CQ for 1 h prior to infection, and cell culture supernatants were collected and assayed for viral yields at 24 hpi. As CQ concentration increased, titers of viral progeny were reduced in CEF cells with CQ treatment compared with those in DMSO-treated cells (Figure 7B). CQ treatment decreases Akt phosphorylation and viral progeny yields in NDV-infected CEF cells, thereby indicating that inhibiting lysosomal acidification reduces Akt phosphorylation and NDV replication.

**Figure 7:** Inhibition of lysosomal acidification reduces Akt phosphorylation and NDV titers CEF cells were preincubated with chloroquine (5–100 μM) for 1 h and then infected with NDV-GM at an MOI of 1. Cell lysates were harvested at 1 hpi for pAkt (Ser 473), and total Akt detection was analyzed by western blot. Cell culture media supernatant aliquots were harvested at 24 hpi to determine virus titers by plaque assay. Data are representative of results of three independent experiments; ns: Not significant, *p < 0.05, **p < 0.01 (*t* test).

### Inhibition the PI3K signaling pathway activated by NDV infection enhances early-stage apoptotic responses

High-titered interferons induced by NDV in infected cells are required for antiviral signaling responses through the activation of STAT3 and antiapoptotic activities [20, 21]. Given that type I and II interferons are known indirect antagonists of programmed cell death, we investigated other possible molecular mechanisms that suppress the induction of programmed cell death. GSK-3β induces apoptosis and is inhibited by Akt phosphorylation [22]. To further verify the role of the PI3K/Akt pathway in the apoptotic signaling response in NDV-infected cells, we preincubated LY294002-infected cells with NDV and analyzed whether the substrate protein, GSK-3β, was associated with the kinase activity of Akt. CEF cells were mock-treated or infected with NDV-GM strain at an MOI of 1 for 12, 18, and 24 h in either the presence or absence of LY294002 (20 μM). Cells were harvested and lysed for western blot with p-Akt and p-GSK-3β antibodies. Pretreating CEF cells with PI3K inhibitor LY294002 reduced the phosphorylation of Akt and GSK-3β at 18 and 24 hpi (Figure 8A). Inhibition of the PI3K/Akt signaling pathway by LY294002 (20 μM) resulted in the cleavage of PARP and caspase 3 in CEF cells at an early phase of NDV infection (Figure 8A), which counters the expression levels of phosphorylated Akt and GSK-3β.

**Figure 8:** Inhibition of PI3K activity results in the apoptosis of CEF cells (**A**) CEF cells were preincubated with the PI3K inhibitor LY294002 (LY) (20 μM) or equal volumes of DMSO for 1 h. They were then infected with NDV-GM at an MOI of 1, and harvested and lysed at 0, 12, 18, and 24 hpi. Specific antibodies were used to assess the phosphorylation of Akt (Ser 473) and GSK-3β, as well as the cleavage of caspase-3 and PARP by western blot. (**B**) CEF cells were pretreated with the specific PI3K inhibitor LY294002 (20 μM) or equal volumes of DMSO for 1 h. After being infected with NDV-GM strain, they were harvested for annexin V apoptosis detection and PI double staining. Then they were analyzed by flow cytometry at 12, 24, and 48 h postinfection (hpi). (**C**) The number of apoptosis cells (*M* ± *SD* of triplicates) are quantified in (B); *p < 0.05, **p < 0.01, ***p < .001 (*t* test).

To further confirm whether PI3K inhibition by LY294002 or wortmannin suppressed the apoptotic signaling responses, we analyzed the number of apoptotic cells using annexin V-FITC and PI double staining assay by flow cytometry. CEF cells were unincubated or pretreated for 1 h with LY294002 (20 μM), infected with NDV infection at an MOI of 1, and then harvested and assayed at 12, 24, and 48 hpi. Cells were infected in the continued presence of LY294002. The NDV-GM strain increased the number of apoptotic cells at 12 hpi (8.5%), and further increased at 24 and 48 hpi (9.8% and 15.8%, respectively) compared with mock-infected cells (Figure 8B, 8C). However, apoptosis increased in CEF cells preincubated with 20 μM LY294002 at 12, 24, and 48 hpi (11.9%, 17.8%, and 24.0%, respectively) compared with untreated NDV-infected cells.

Overall, the inhibition of the PI3K signaling pathway diminishes the onset of premature NDV-triggered apoptosis at an early phase of infection.

### Inhibition of apoptosis enhances cell survival upon NDV infection

As described above, the activation of the PI3K/Akt signaling pathway in NDV-infected cells results in antiapoptotic effects. To test the effect of pan caspase inhibitor and apoptosis on NDV-induced cell survival, we preincubated CEF cells for 1 h with increasing concentrations of pan caspase inhibitor ZVAD-FMK (10, 20, 30, and 40 μM) in either the absence or presence of LY294002 (20 μM). They were infected with the NDV-GM strain at an MOI of 1. At 1 hpi, the infected cells were harvested and lysed for western blot with the p-Akt antibody. Compared to the NDV-infected cells in the absence of the PI3K inhibitor, cells pretreated with ZVAD-FMK of NDV-infected cells in the presence of LY294002 altered overall Akt levels and increased the level of phosphorylated Akt in a dose-dependent manner (Figure 9A).

**Figure 9:** Pharmacological inhibition of apoptosis enhances NDV-triggered cell survival CEF cells were pretreated with ZVAD-FMK (10, 20, 30, and 40 μM) for 1 h with or without LY294002 (20 μM) prior to infection with NDV-GM at an MOI of 1. (**A**) At 1 hpi, cells were harvested and lysed for western blot using the pAkt (Ser 473) and total Akt antibody. (**B**) At 24 hpi, cell lysates were harvested and subjected to western blot with caspase 3 and PARP antibodies. (**C**) At 24 hpi, cell viability was measured by MTT assay; *p < .05, **p < .01 (*t* test). (**D**) At 24 hpi, the number of apoptotic cells were calculated by flow cytometry using Annexin V-FITC/PI Apoptosis Detection Kit; *p < .05 (*t* test).

To further investigate whether inhibiting apoptosis promotes host cell survival, we examined the cleavage of host proteins associated with hallmark features of apoptosis, caspase 3 and PARP. CEF cells were preincubated for 1 h with increasing concentrations of the pan caspase inhibitor ZVAD-FMK (10, 20, 30, and 40 μM) in either the absence or presence of LY294002 (20 μM) before their infection with NDV-GM strain at an MOI of 1. Infected cells were harvested and lysed at 24 hpi for western blot with cleaved-caspase 3 and -PARP antibodies. Cleavage of caspase-3 and PARP by the pan caspase inhibitor ZVAD-FMK due to the inhibition of the survival pathway by LY294002 was inhibited in a dose-dependent manner (Figure 9B).

As described above, cell viability and the number of apoptotic cells after pretreatment with increasing concentrations ZVAD-FMK in either the absence or presence of LY294002 (20 μM) at 24 hpi were measured. Lower concentrations of ZVAD-FMK (10 and 20 μM) displayed no evident antiapoptotic effects in CEF cells; however, the high concentration of ZVAD-FMK (40 μM) increased cell viability in the presence of LY294002 (Figure 9C). In addition, antiapoptotic effects induced upon incubation with ZVAD-FMK not only increased cell viability, but also decreased the number of apoptotic cells (Figure 9D).

### Inhibition of PI3K activity and apoptosis can prevent NDV replication

Specific PI3K inhibitor LY294002- or wortmannin-induced inhibition of viral protein expression might be due to accelerated apoptosis signals in NDV-infected cells. To explore this, CEF cells were incubated for 1 h with pan caspase inhibitor ZVAD-FMK (40 μM) in either the absence or presence of LY294002 (20 μM) and infected with the NDV-GM strain at an MOI of 1. At 48 hpi, cells were harvested for western blot with the NDV-P protein antibody, and for a cell viability count. Treatment with ZVAD-FMK in the presence of LY294002 blocked cell death in NDV-infected CEF cells (Figure 10A). In NDV-infected cells, pretreatment with pan caspase inhibitor ZVAD-FMK in the presence of LY294002 results in a 13.7% decrease in the apoptotic cell count compared to pretreatment with LY294002 alone (Figure 10B). As expected, pretreatment with LY294002 (20 μM) resulted in a decrease in the NDV-P protein expression level compared to untreated NDV-infected cells (Figure 10C). However, inhibition of apoptotic signals by the pan caspase inhibitor ZVAD-FMK (40 μM) reversed the inhibitor effect of LY294002 on NDV-P protein expression. Similar results were obtained using wortmannin (data not shown). The antiapoptotic PI3K activity exerted during NDV replication is a caspase-dependent event, and consolidates the functional interaction of the PI3K/Akt signaling pathway and apoptosis during NDV infection.

**Figure 10:** PI3K signaling pathway and apoptosis are simultaneously involved in NDV replication CEF cells were preincubated with the pan caspase inhibitor ZVAD-FMK (40 μM) for 1 h, with or without PI3K inhibitor LY294002 (LY) (20 μM) prior to infection with NDV-GM at an MOI of 1 for 48 h. (**A**) Cell death was analyzed under microscope and by MTT assay. (**B**) The number of apoptotic cells was calculated by flow cytometry using Annexin V-FITC/PI Apoptosis Detection Kit. *p < .05, ***p < .001 (*t* test). (**C**) Cell lysates were harvested and subjected to western blot using the anti-NDV P antibody. *p < .05 (*t* test).

## DISCUSSION

Viral infection results in the activation of a variety of intracellular signaling pathways, including PI3K/Akt. These pathways are partly required to mount an antiviral response to infection, yet can also be exploited by the virus to promote its replication [23]. We demonstrated that NDV-infected CEF cells could activate Akt phosphorylation as early as 15 mpi and peak at 60 mpi. However, that activation phenomenon was transient and no longer visible at 24 hpi (Figure 1), thereby suggesting that NDV's activation of the PI3K/Akt signaling pathway does not depend on virus replication. Inhibition of the PI3K/Akt signaling pathway can decrease viral progeny yields (Figure 5B), which suggests the PI3K/Akt signaling pathway also promotes NDV replication. Inhibition of the PI3K/Akt signaling pathway also results in the cleavage of caspase 3 and PARP, as well as increases apoptotic cells per annexin V and PI double staining assay but not GSK-3β phosphorylation (Figure 8). This demonstrates that NDV-infected chicken cells enhance the apoptotic response during the early phase of infection. Furthermore, inhibition of PI3K/Akt activity by an enhanced apoptosis signal response could be largely reversed by the pan caspase inhibitor ZVAD-FMK, thereby indicating that the PI3K/Akt signaling pathway could promote cellular survival.

Many viruses can induce the activation of PI3K/Akt signaling in infected cells [13, 24, 25]. We applied specific PI3K inhibitor LY294002 or wortmannin to NDV-infected CEF cells, and the resulting Akt phosphorylation levels decreased (Figure 2). This indicates that activating Akt in NDV-infected CEF cells depends on PI3K in the early stage of viral infection. We also observed the activation of Akt phosphorylation by UV-inactivated NDV in CEF cells (Figure 4), which implies that activating the PI3K/Akt signaling pathway does not require viral replication. This suggests a possible role of the interaction of NDV and its receptors, and indicates the involvement of virus receptor attachment in viral entry and budding.

Regarding the course of viral entry into host cells, several viruses prompt PI3K/Akt activation during the early stages of viral infection without viral replication [13, 24, 26–28]. At early stages of infection, PI3K/Akt activation is triggered by intracellular viral protein synthesis and viral attachment [26], [28], [29], and by viral entry and endosomal sorting [27, 30]. During late stages of infection, PI3K/Akt signaling regulates viral assembly and release [31, 32]. We observed Akt phosphorylation in NDV-infected CEF and DF-1cells during the early stage of viral infection (15 mpi–12 hpi), which coincides with NDV entry into host cells by clathrin-mediated endocytosis. To further examine whether Akt phosphorylation occurred after virus attachment to the host cell membrane, we used methyl-β-cyclodextrin and chlorpromazine, a pharmacological inhibitor of clathrin-mediated endocytosis, which decreased the virus particles that invaded the host's infected cells (Figure 3). Our results show that early activation of the PI3K/Akt signaling pathway induced by NDV is induced by endocytosis.

Several viruses activate the PI3K/Akt signaling pathway at early stages of viral infection [13, 25, 33, 34], which further promotes viral replication and host cell survival. In our study, inhibition the PI3K/Akt signaling pathway reduced viral replication (Figure 5) and viral protein synthesis (Figure 10C), thereby suggesting that activating the PI3K/Akt signaling pathway can promote virus replication. PI3K supports the viral life cycle, such as in viral entry and budding, and inhibition of PI3K activity can decrease virus proliferation and gene synthesis [13, 35, 36]. Our results indicate that inhibiting PI3K activity reduces viral protein replication (Figure 6), thereby suggesting that PI3K activity stimulates NDV's infection cycle.

Chloroquine inhibits the activation of PI3K and transcription factor NF-κB induced by respiratory syncytial virus, which in turns delays the antiapoptotic effect by preventing neutrophil and eosinophil apoptosis [14]. Likewise in our study, Akt phosphorylation and viral protein synthesis were reduced by pretreatment with lysosomotropic amine chloroquine (Figure 7), thus suggesting that PI3K activation is required for endolysosomal internalization.

During the early stages of viral infection, many viruses induce PI3K activation, which in turns activates different antiapoptotic factors [13, 14, 37–40], including Akt and GSK3β, to support viral replication by preventing apoptosis in infected cells. The PI3K/Akt signaling pathway might provide new opportunities for novel antiviral targets, especially for emerging infectious viruses such as Zika virus. GSK3β has been identified as a physiological target of Akt [22]. During short-term infection, PI3K/Akt inhibition in NDV-infected CEF cells decreases GSK-3β phosphorylation compared to NDV-infected cells alone (Figure 8A), yet increases the cleavages of caspase-3, PARP, and the number of apoptotic cells (Figures 8, Figure 9). The PI3K/Akt signaling pathway suppresses apoptosis for cell survival by preventing the onset of premature NDV-induced caspase activation and apoptosis early on in viral infection.

Triggered by many viruses, the PI3K/Akt signaling pathway maintains cell viability and proliferation by interfering with pro-apoptotic signaling response, which in turn activates downstream transcription factors and promotes virus replication [12, 41]. We found PI3K/Akt inhibition triggered by NDV in CEF cells increased the cleavage of caspase 3 and PARP, as well as the number of apoptosis cells during the early phase of infection. This indicates the PI3K molecule might have an antiapoptotic signaling role. Our results also demonstrate that pan caspase inhibitor ZVAD-FMK reduces the cleavage of caspase 3 and PARP and the number of apoptosis cells associated with PI3K inhibitor. ZVAD-FMK also increases Akt phosphorylation and cell viability (Figure 9). Those results demonstrate that NDV-induced PI3K/Akt activation in a host's infected cells prolongs cell survival, and thereby facilitates viral replication.

Our results clearly show that NDV can transiently activate the PI3K/Akt signaling pathway during the early stage of infection, which in turn inhibits the onset of premature NDV-induced apoptosis, and promotes both cell survival and viral replication in infected cells. Our data therefore indicate new opportunities for unraveling novel targets of the PI3K/Akt pathway to develop a potential antiviral drug against NDV.

## MATERIALS AND METHODS

### Ethics statement

This study was conducted with the approval of the South China Agricultural University Experimental Animal Welfare Ethics Committee (permit no. 2015–03).

### Viruses and cells

Three NDV strains – GM (genotype VII), F48E9 (genotype IX), and La Sota (genotype II) – were obtained from South China Agricultural University (Guangzhou, China), plaque-purified, and grown in the allantoic cavity of 10-d old embryonated chicken eggs (Chinese Academy of Agriculture, Beijing, China) at 37°C, as previously described [42, 43]. Allantoic fluid was harvested 48 h after inoculation and stored at −80°C for further characterization. Chicken embryo fibroblast (CEF) primary cells were made from 10-d old specific-pathogen-free (SPF)-embryonated chicken eggs, also as previously described [44]. To obtain the replication-incomplete NDV-GM strain, fresh infected allantoic fluid (5 mL) was irradiated with ultraviolet (UV) light for 30 min. The absence of virus infectivity following UV treatment was confirmed by the lack of replication in CEF cells and 10-d-old SPF-embryonated chicken eggs. Chicken fibroblast cell line DF-1 (CRL-12203) was purchased from the American Type Culture Collection. CEF and DF-1 cells were grown in Dulbecco's modified Eagle medium (DMEM) (Invitrogen, Carlsbad, CA, USA) supplemented with 5% fetal bovine serum (Gibco, Thermo Scientific, Waltham, MA, USA), 100 U/mL penicillin, and 100 μg/mL streptomycin. They were grown overnight at 37°C with 5% CO_2_ until they reached approximately 80% confluence.

### Antibodies and reagents

Specific PI3K inhibitors LY294002 and wortmannin were provided by Calbiochem (Billerica, MA, USA). Chlorpromazine (Chl), chloroquine (CQ), methyl β-cyclodextrin (MβCD), Akt, pAkt-473, and anti-GAPDH antibodies were purchased from Sigma–Aldrich (Shanghai, China). Cleaved caspase-3, cleaved PARP, and phosphospecific glycogen synthase kinase-3β (GSK-3β) and its antibodies were obtained from Cell Signaling Technology (Beverly, MA, USA). The polyclonal antibody against NDV P protein was provided by South China Agricultural University. Infrared dye 680 (i.e., goat anti-rabbit IgG) and 800CW (i.e., goat anti-mouse IgG) were purchased from LI-COR (Lincoln, NE, USA), and pan caspase inhibitor ZVAD-FMK from InvivoGen (Carlsbad, CA, USA).

### Virus infectivity assay

For infection, cells were washed with phosphate-buffered saline (PBS) and incubated with the virus at the indicated multiplicities of infection (MOI) diluted in DMEM for 60 min at 39°C. The inoculum was aspirated, and the cells were incubated with either minimal essential medium or DMEM containing 100 U/ml penicillin and 0.1 mg/ml streptomycin. All media were supplemented with 10% heat-inactivated fetal bovine serum (Invitrogen).

### Cell viability assay (MTT assay)

Cell viability in the presence or absence of different inhibitors or dimethyl sulfoxide (DMSO) was measured by a 3-[4, 5-dimethylthiazol-2-yl]-2, 5 diphenyltetrazolium bromide (MTT)-based assay (Cell Growth Determination Kit, Sigma–Aldrich) in accordance with the manufacturer's protocol. CEF or DF-1 cells were seeded into 96-well plates and pretreated with different inhibitors or DMSO for various lengths of time. After each incubation period, 10 μL of MTT labeling mixture was added to each well, and cells were incubated at 37°C for 4 h. Absorbance was measured by an enzyme-linked immunosorbent assay reader at a wavelength of 490 nm. Data represent the average of at least three independent experiments.

### Western blot

Cells were rinsed with PBS and lysed with radioimmune precipitation assay buffer (50 mM tris-HCl [pH 7.4], 150 mM NaCl, 0.1% SDS, 0.5% sodium deoxycholate, 1%Triton X-100, 1 mM PMSF). Following sonication, cell lysates were subjected to centrifugation to remove cell debris. An aliquot of the supernatant containing 20 μg of protein was used for gel electrophoresis, and transferred onto nitrocellulose membranes (Roche, Manheim, Germany) using the iBlot Gel Transfer Device (Bio-Rad, Redmond, WA,USA). Membranes were blocked with 5% BSA for 1 h at 37°C, and incubated overnight at 4°C with the primary antibody. After three washes with TBS containing 0.5% Tween 20 (TBST), membranes were incubated at 37°C for 1 h in infrared dye 680 or 800 (1:5,000) diluted in TBST as the secondary antibody. Once membranes were washed three times in TBST again, they were visualized and analyzed with an Odyssey infrared imaging system (LI-COR).

### Flow cytometry

Apoptosis was detected by flow cytometry using Annexin V-FITC/PI Apoptosis Detection Kit (Sigma–Aldrich), following the manufacturer's instructions. 10,000 CEF or DF-1 cells were pretreated with LY294002 (20 μM) or DMSO for 1 h and infected with GM at an MOI of 1. Cells were harvested, washed with ice cold PBS three times, centrifuged, and suspended with 500 μL 10X binding buffer. They were incubated with 10 uL annexin V per test for 10 min at room temperature. Later, 5 μL propidium iodide (PI) was added per test, and the product incubated for 5 min. The final cells were qualified and analyzed with a FC500 flow cytometer (Beckman Coulter, Brea, CA, USA). Data were determined as the average percentage of apoptotic cells in three independent experiments.

### Statistical analysis

Results are presented as *M* ± *SD* or *SE*. Statistical comparisons were calculated by using Student's *t* test, and differences between groups were considered significant if *p* < .05.

## References

[1] Elankumaran S, Rockemann D, Samal SK (2006). Newcastle disease virus exerts oncolysis by both intrinsic and extrinsic caspase-dependent pathways of cell death. J Virol.

[2] Sinkovics JG, Horvath JC (2000). Newcastle disease virus (NDV): brief history of its oncolytic strains. J Clin Virol.

[3] Alexander DJ (2000). Newcastle disease and other avian paramyxoviruses. Rev Sci Tech.

[4] Steward M, Vipond IB, Millar NS, Emmerson PT (1993). RNA editing in Newcastle disease virus. J Gen Virol.

[5] Park MS, Shaw ML, Munoz-Jordan J, Cros JF, Nakaya T, Bouvier N, Palese P, Garcia-Sastre A, Basler CF (2003). Newcastle disease virus (NDV)-based assay demonstrates interferon-antagonist activity for the NDV V protein and the Nipah virus V, W, and C proteins. J Virol.

[6] Eckert DM, Kim PS (2001). Mechanisms of viral membrane fusion and its inhibition. Annu Rev Biochem.

[7] Cantin C, Holguera J, Ferreira L, Villar E, Munoz-Barroso I (2007). Newcastle disease virus may enter cells by caveolae-mediated endocytosis. J Gen Virol.

[8] K San Roman, Villar E, Munoz-Barroso I (1999). Acidic pH enhancement of the fusion of Newcastle disease virus with cultured cells. Virology.

[9] Gingras AC, Kennedy SG, O'Leary MA, Sonenberg N, Hay N (1998). 4E-BP1, a repressor of mRNA translation, is phosphorylated and inactivated by the Akt(PKB) signaling pathway. Genes Dev.

[10] Manning BD, Cantley LC (2007). AKT/PKB signaling: navigating downstream. Cell.

[11] Wullschleger S, Loewith R, Hall MN (2006). TOR signaling in growth and metabolism. Cell.

[12] Diehl N, Schaal H (2013). Make yourself at home: viral hijacking of the PI3K/Akt signaling pathway. Viruses.

[13] Ehrhardt C, Wolff T, Pleschka S, Planz O, Beermann W, Bode JG, Schmolke M, Ludwig S (2007). Influenza A virus NS1 protein activates the PI3K/Akt pathway to mediate antiapoptotic signaling responses. J Virol.

[14] Lindemans CA, Coffer PJ, Schellens IM, de Graaff PM, Kimpen JL, Koenderman L (2006). Respiratory syncytial virus inhibits granulocyte apoptosis through a phosphatidylinositol 3-kinase and NF-kappaB-dependent mechanism. J Immunol.

[15] Guo H, Zhou T, Jiang D, Cuconati A, Xiao GH, Block TM, Guo JT (2007). Regulation of hepatitis B virus replication by the phosphatidylinositol 3-kinase-akt signal transduction pathway. J Virol.

[16] Rejman J, Bragonzi A, Conese M (2005). Role of clathrin- and caveolae-mediated endocytosis in gene transfer mediated by lipo- and polyplexes. Mol Ther.

[17] Rodal SK, Skretting G, Garred O, Vilhardt F, van Deurs B, Sandvig K (1999). Extraction of cholesterol with methyl-beta-cyclodextrin perturbs formation of clathrin-coated endocytic vesicles. Mol Biol Cell.

[18] Diebold SS, Kaisho T, Hemmi H, Akira S, Reis e Sousa C (2004). Innate antiviral responses by means of TLR7-mediated recognition of single-stranded RNA. Science.

[19] Lee J, Chuang TH, Redecke V, She L, Pitha PM, Carson DA, Raz E, Cottam HB (2003). Molecular basis for the immunostimulatory activity of guanine nucleoside analogs: activation of Toll-like receptor 7. Proc Natl Acad Sci USA.

[20] Wheelock EF (1966). Virus replication and high-titered interferon production in human leukocyte cultures inoculated with Newcastle disease virus. J Bacteriol.

[21] Youngner JS, Scott AW, Hallum JV, Stinebring WR (1966). Interferon production by inactivated Newcastle disease virus in cell cultures and in mice. J Bacteriol.

[22] Pap M, Cooper GM (1998). Role of glycogen synthase kinase-3 in the phosphatidylinositol 3-Kinase/Akt cell survival pathway. J Biol Chem.

[23] Deane JA, Fruman DA (2004). Phosphoinositide 3-kinase: diverse roles in immune cell activation. Annu Rev Immunol.

[24] Ehrhardt C, Ludwig S (2009). A new player in a deadly game: influenza viruses and the PI3K/Akt signalling pathway. Cell Microbiol.

[25] Ehrhardt C, Wolff T, Ludwig S (2007). Activation of phosphatidylinositol 3-kinase signaling by the nonstructural NS1 protein is not conserved among type A, B influenza viruses. J Virol.

[26] Saeed MF, Kolokoltsov AA, Freiberg AN, Holbrook MR, Davey RA (2008). Phosphoinositide-3 kinase-Akt pathway controls cellular entry of Ebola virus. PLoS Pathog.

[27] Lau C, Wang X, Song L, North M, Wiehler S, Proud D, Chow CW (2008). Syk associates with clathrin and mediates phosphatidylinositol 3-kinase activation during human rhinovirus internalization. J Immunol.

[28] Wong WR, Chen YY, Yang SM, Chen YL, Horng JT (2005). Phosphorylation of PI3K/Akt and MAPK/ERK in an early entry step of enterovirus 71. Life Sci.

[29] Linero FN, Scolaro LA (2009). Participation of the phosphatidylinositol 3-kinase/Akt pathway in Junin virus replication in vitro. Virus Res.

[30] Marjuki H, Gornitzky A, Marathe BM, Ilyushina NA, Aldridge JR, Desai G, Webby RJ, Webster RG (2011). Influenza A virus-induced early activation of ERK and PI3K mediates V-ATPase-dependent intracellular pH change required for fusion. Cell Microbiol.

[31] Carsillo M, Kim D, Niewiesk S (2010). Role of AKT kinase in measles virus replication. J Virol.

[32] Jeffree CE, Brown G, Aitken J, Su-Yin DY, Tan BH, Sugrue RJ (2007). Ultrastructural analysis of the interaction between F-actin and respiratory syncytial virus during virus assembly. Virology.

[33] Soares JA, Leite FG, Andrade LG, Torres AA, De Sousa LP, Barcelos LS, Teixeira MM, Ferreira PC, Kroon EG, Souto-Padron T, Bonjardim CA (2009). Activation of the PI3K/Akt pathway early during vaccinia and cowpox virus infections is required for both host survival and viral replication. J Virol.

[34] Rahaus M, Desloges N, Wolff MH (2007). Varicella-zoster virus requires a functional PI3K/Akt/GSK-3alpha/beta signaling cascade for efficient replication. Cell Signal.

[35] Feng SZ, Cao WS, Liao M (2011). The PI3K/Akt pathway is involved in early infection of some exogenous avian leukosis viruses. J Gen Virol.

[36] Urata S, Ngo N, de la Torre JC (2012). The PI3K/Akt pathway contributes to arenavirus budding. J Virol.

[37] Esfandiarei M, Luo H, Yanagawa B, Suarez A, Dabiri D, Zhang J, McManus BM (2004). Protein kinase B/Akt regulates coxsackievirus B3 replication through a mechanism which is not caspase dependent. J Virol.

[38] Peters K, Chattopadhyay S, Sen GC (2008). IRF-3 activation by Sendai virus infection is required for cellular apoptosis and avoidance of persistence. J Virol.

[39] Prejean C, Sarma T, Kurnasov O, Usacheva A, Hemmings B, Cantley L, Fruman DA, Morrison LA, Buller RM, Colamonici OR (2001). Phosphatidylinositol 3-kinase confers resistance to encephalomyocarditis and herpes simplex virus-induced cell death through the activation of distinct downstream effectors. J Immunol.

[40] Wei L, Zhu S, Wang J, Liu J (2012). Activation of the phosphatidylinositol 3-kinase/Akt signaling pathway during porcine circovirus type 2 infection facilitates cell survival and viral replication. J Virol.

[41] Datta SR, Brunet A, Greenberg ME (1999). Cellular survival: a play in three Akts. Genes Dev.

[42] Kang Y, Li Y, Yuan R, Feng M, Xiang B, Sun M, Xie P, Tan Y, Ren T (2015). Host Innate Immune Responses of Ducks Infected with Newcastle Disease Viruses of Different Pathogenicities. Front Microbiol.

[43] Kang Y, Xiang B, Yuan R, Zhao X, Feng M, Gao P, Li Y, Ning Z, Ren T (2016). Phylogenetic and Pathotypic Characterization of Newcastle Disease Viruses Circulating in South China and Transmission in Different Birds. Front Microbiol.

[44] Kang Y, Feng M, Zhao X, Dai X, Xiang B, Gao P, Li Y, Ren T (2016). Newcastle disease virus infection in chicken embryonic fibroblasts but not duck embryonic fibroblasts is associated with elevated host innate immune response. Virol J.

